This article has been retracted.

# Evaluation of fluorinated phospholipid analogs: A study on ADMET profiles, molecular docking and dynamics simulation in anticancer therapy

**DOI:** 10.1016/j.heliyon.2025.e41739

**Published:** 2025-01-10

**Authors:** Saqib Ishaq, Obaid Habib, Abdul Aziz, Raheel Tahir, Hira Mushtaq, Said Hassan, Sarah Sarwar, Mohammad S. Mubarak, Ajaz Ahmad, Amin Ullah

**Affiliations:** a Guangdong Provincial Key Laboratory of System Biology and Synthetics Biology for Urogenital Tumors, School of Basic Medicine, Shenzhen University Medical School, Shenzhen University (SZU), Guangdong, China; b Department of Computer Sciences and Bioinformatics, Khushal Khan Khattak University, Karak, Khyber Pakhtunkhwa, Pakistan; c Department of Biotechnology and Genetic Engineering, Kohat University of Science and Technology (KUST), Kohat, KP, Pakistan; d Centre of Biotechnology and Microbiology, University of Peshawar, 25000, Peshawar, Pakistan; e Institute of Biotechnology and Microbiology, Bacha Khan University Charsada, 24550, Charsada, Pakistan; f Department of Biochemistry, Shaheed Benazir Bhutto Women University Peshawar, 25000, Peshawar, Pakistan; g Department of Chemistry, Indiana University Bloomington, 47405, Bloomington, USA; h Department of Chemistry, University of Jordan, Amman, 11942, Jordan; i Department of Clinical Pharmacy, College of Pharmacy, King Saud University, 11451, Riyadh, Saudi Arabia; j Department of Allied Health Sciences, Molecular Biology Lab, Iqra National University (INU) Peshawar, 25000, Peshawar, Pakistan

**Keywords:** ADMET properties, Toxicity, Admetsar, CLC-Pred, Molecular docking, MD simulation

## Abstract

Fluorinated phospholipid analogs Edelfosine and Ilmofosine drug reveal expressive potential as antineoplastic factors though targeted interaction with heat shock protein (HSP70KDa1A), an essential mediator in cancer pathophysiology. Using evolved computational approaches, this research evaluated their ADMET (absorption, distribution, metabolism, excretion and toxicity) profiles receptor binding affinities and molecular dynamics. Molecular docking discernible vigorous interactions with Edelfosine drug displaying greater binding stability and consistent hydrogen bonding as confirmed by 100 ns molecular dynamics simulations. Comparative interpretation emphasized Edelfosine drug enhanced pharmacokinetic properties depicted by lower RMSD values, stable solvent-accessible surface area and reduced structural fluctuations relative to Ilmofosine drug. Functional annotation and phylogenetic investigation affirmed the evolutionary conservation and pivotal biological function of heat shock protein (HSP70KDa1A). These findings position Edelfosine drug as a promising candidate for targeted cancer therapy appropriated further experimental validation to elucidate its mechanisms of action and therapeutic efficacy.

## 1 Introduction

The defining characteristic of cancer is uncontrolled cellular proliferation within the human body. These abnormal cells, frequently referred to as cancer cells, carcinomas, or tumor cells, have the capacity to penetrate and endanger the integrity of healthy, normal tissues. The term “cancer” refers to a wide range of illnesses, each of which is named after the tissue from where it originated, such as breast carcinoma, pulmonary malignancy and colorectal neoplasia [1]. The causes of cancer are diverse and involve a complex interaction of variables, including some unrecognized ones. Environmental variables, dietary habits and genetic predisposition may all have an impact on how this condition develops. A variety of factors, such as inherited characteristics, exposure to ionizing radiation, chemical agents, dietary habits, virus infections and psychological stressors often come together to cause cancer. Additionally, increasing aged is recognized as a significant risk factor for the occurrence of cancer [2,3].

Recent studies indicate a rising trend in cancer incidence, particularly in Asia and emerging nations. Studies have shown that as compared to western counterparts, several Asian countries have higher rates of various cancer kinds, with lung and colorectal cancer being two prominent instances. At the moment, Asia accounts for 48 % of new cancer diagnoses worldwide with china accounting for over half of these cases [4]. Moreover, Asia accounts for 55 % of the global mortality rates for cancer-related deaths, making it the region worst hit. Within the next 20 years, recent studies predict a rise in cancer incidence and fatality rates throughout Asian countries. Previous worldwide study has supported the idea that cancer prevalence varies depending on a variety of variables, including age demographics, gender distribution, location, and the economic standing of the individual countries [5,6].

In Pakistan, breast cancer is the most frequently diagnosed cancer in women (n = 34,038, 40.2 %), followed in descending order by cancers of the mouth, cervix, uterine, ovary and esophagus (n = 2,718, 3.2 %). With a 1.2 % contribution and 1,029 new cases per year, lung cancer was ranked 12th on the list [7]. Women in Pakistan lost their lives to cancer in 2012, resulting in 52,664 fatalities overall, or 144 on daily. Breast cancer was the leading cause of mortality, contributing to 16,232 deaths (30.8 %). Following it were cancers of the mouth, cervix, ovary and esophagus, which caused 6.1 %, 5.5 %, and 5.2 % of fatalities, respectively. Those who are older have a greatly increased risk of having lung cancer. Less than 2 % of lung cancer diagnoses in people under 45 happen in people who are 65 years or older, who make up around two-thirds of all cases. The average age at diagnosis for lung cancer is almost 70 years old. Notably, the average lifetime of men in Pakistan is 65.5 years, and men often develop lung cancer at the age of 63, indicating the diseases link to advanced age. The average life expectancy in Pakistan is lower than the average age at which lung cancer is most likely to develop, with a peak age of occurrence of 70 years. While the average life expectancy for women in Pakistan is 67.5 years, the peak age for lung cancer incidence is 68.5 years [7]. The majority of individuals with pancreatic cancer receive a diagnosis when the disease is well advanced, which results in an extremely poor survival rate of just 4–6 months. The only curative option is surgical tumor removal, which is frequently followed by adjuvant chemotherapy using drugs like 5-fluorouracil and gemcitabine. Unfortunately, less than 20 % of patients respond to the popular medicine gemcitabine, which has prompted ongoing clinical trials to find pharmacological combinations with synergistic effects for better therapeutic results [8]. The endoplasmic reticulum (ER), which is in control of regulating the processes of protein folding and modification, is essential for preserving cellular viability and functionality. A variety of transcriptional, metabolic and oncogenic alterations in tumor cells triggers abnormal endoplasmic reticulum action, which results in misfolded proteins in cancerous cells. Endoplasmic reticulum (ER) stress that is prolonged and excessive can result in the buildup of misfolded proteins within endoplasmic reticulum the (ER) lumen [9]. The unfolded protein response (UPR), which seeks to reestablish normal endoplasmic reticulum (ER) functions is triggered by this buildup. The unfolded protein responses (UPR's) initially cytoprotective functions, however, can change into the ability to promote cell death when the endoplasmic reticulum (ER) stress is ongoing. This can cause endoplasmic reticulum (ER) dependent apoptotic pathways to be activated, ultimately leading to cell death. Endoplasmic reticulum (ER) stress can also contribute to the development of pancreatic cancer. Studies have revealed that the three main mechanisms of endoplasmic reticulum (ER) stress-induced apoptosis in pancreatic cancer cells include overexpression of the transcription factor CHOP/GADD153, activation of JNK, and activation of caspase-12 in murine systems or caspase-4 in human cells [10]. Additionally, research suggests that targeting the endoplasmic reticulum (ER) stress pathway through the inhibition of specific molecules, such as IRE1α, may have therapeutic potential in treating pancreatic cancer [11]. However, more research is needed to fully understand the role of endoplasmic reticulum (ER) stress in the development and progression of pancreatic cancer and to determine the most effective therapeutic strategies. Recent discoveries have illuminate the potential of fluorinated phospholipids in cancer therapy due to their ability to increase the bioavailability, lipophilicity and metabolic stability of drug molecules. Studies have demonstrate that fluorination of alkylphosphocholine analogs, including Edelfosine and Ilmofosine enhances their pharmacokinetic profiles and increases their selective cytotoxicity toward cancer cells [12]. Additionally, targeting heat shock proteins (HSP HSP70KDa1A) has appeared as a promising therapeutic approach. These proteins play critical characteristics in tumor cell survival under stress conditions making them key targets for anticancer drug development. Recent investigation have concentrated on inhibiting heat shock proteins to influence apoptosis in cancer cells, demonstrating the effectiveness of combined strategies involving fluorinated phospholipids and heat shock protein inhibition in enhancing therapeutic consequences [13].

Alkyl-lysophospholipid analogs (ALPs) are a large variety of synthetic lipids that lead to apoptosis in a range of tumor cells [14]. The anticancer drugs Edelfosine and Miltefosine, which affect the endoplasmic reticulum, are among the most effective Alkyl-lysophospholipid analogs (ALPs) in alleviating human pancreatic cancer cells. The drugs have high uptake by pancreatic cancer cells, which significantly induces malignant cell apoptosis via caspase and mitochondria. However, their metabolic instability, lack of selectivity, and high gastrointestinal toxicity have led to investigations of alternatives [15]. The selectivity and stability of macromolecules or compartments can be altered through partial or complete fluorination of alkyl chains. The fluorination of alkyl-lysophospholipids (ALPs) is a fundamental region of research due to the known ability of fluorine atoms to increase the metabolic homeostasis, bioavailability and lipophilicity of drug molecules. Integrating fluorine into alkyllysophospholipid analogs (ALPs) may conduct to progressive therapeutical characteristics, constituting this strategy relevant for the improvement of highly competent prescription, specifically in overcoming impediment procedure and improving therapeutic efficiency. The effect of fluorination on the anticancer and ADMET profiles of anticancer drugs Miltefosine, Edelfosine, and Ilmofosine will be investigated in the proposed study using in silico tools. Researchers have applied molecular docking in determining the potential alkyl-phosphocholine. However, no systematic study has been undertaken so far.

## 2 Materials and methods

### 2.1 Materials

Docking represent a computational technique used to assess the interaction between candidate drug ligand and protein, enabling the prediction of the most favorable binding orientation for two molecules to form stable complex. Docking serves as a method for forecasting the affinity and binding activity of small molecule to their respective protein target through the utilization of scoring function. The sensitivity of docking calculation with respect to the input drug geometry highlights that minor alteration in the ligand conformation can results in significant variation in both the geometries and scores of the docking poses. In this study we utilized the web based online molecular docking program known as 1-click docking (https://mcule.com/apps/1-click-docking/). To assessed drug likeness using the binding property explore and conducted ADMET profiling using the admetSAR program. The program successfully computed the crucial docking parameters yielding satisfactory results. It furnished with comprehensive docking outcomes, enabling us to assess the efficacy of test ligand.

### 2.2 ADMET profiling and toxicity assessment of drug candidates

The ADMET property of a compound encompass with its absorption, distribution, metabolism, excretion, and toxicity within the human body. ADMET comprising the pharmacokinetic and antineoplastic profile of a drug molecule, play a pivotal role in assessing its pharmacodynamics activities [16]. Currently a plethora of online and offline software program are accessible to aid in forecasting the behavior of the drug candidate. In this investigation we employed the admetSAR [17] prediction tool (http://lmmd.ecust.edu.cn:8000/) and swissADME [18]. To obtained the toxicity information for each ADMET profile from CLC-pred [19] (http://www.way2drug.com/cell-line/).

### 2.3 Protein receptor selection

The heat shock protein (hsp70KDa 1A) was retrieved with the following identifier (UNIPROT ACCESSION ID: P0DMV8: PDB ID: 2e8a) using the 1-click docking server (https://mcule.com/apps/1-click-docking/). Due to its crystal structure represent a pharmacological target for the development of potential drugs such as (Edelfosine, Ilmofosine) for treatment to which heat shock protein (hsp70KDa1A) was chosen for modeling studies. The 1-click docking server was employed to identify the target containing an active binding site for the drug molecules.

### 2.4 Identification and design of drug ligand

To identify the canonical simplified molecular input line entry system (SMILEs) analog of such as Edelfosine and Ilmofosine from PubChem database (https://pubchem.ncbi.nlm.nih.gov//). Their structure were freshly designed using ChemDraw software [20]. Subsequently, the drug ligand compound obtained by importing their fluorinated from ChemDraw.

### 2.5 Molecular docking

1-click docking accessible at (https://mcule.com/apps/1-click-docking//) is a web based user-friendly interface designed to streamline every aspect of molecular docking, including drug ligand and protein configuration. The protein was accomplished from the Protein Data Bank (PDB) and prepared by eliminate water molecules, expanding hydrogen atoms and optimizing its structure. Drug ligands were prepared by provoke their 3D structures and attribute hydrogenation at physiological pH. The active binding site was distinguish based on key functional residues from the literature and centered in the docking grid, establish detailed binding pose predictions. The binding site was restricted based on active site residues, with docking parameters including as exhaustiveness optimized and grid size for accurate investigation. Docking was conveyed out with flexible ligands and a rigid protein. This platform accommodate various software design, facilitation dynamic and reliable docking calculations with customizable parameters for ligand and receptor setup. Additionally, it offer provide users complete autonomy in configuring specific parameters for ligand and receptor setup as well as conducting docking calculation. To improve the accuracy of our outcomes, we operated verify tests, including a re-docking evaluation, utilizing the 1-Click Docking server for molecular docking. It enable user to perform highly efficient and reliable docking calculation by integrating numerous well-known software program used in In-Silico chemistry and comprehensive web service.

### 2.6 Integrated functional annotation and phylogenetic analysis

The Structural and functional annotation of heat shock protein (hsp70KDa 1A) aimed to identifying it's structural and functional attributes implying Blast2GO typically involve a series of sequential steps. Blast2GO [21] is widely used designed to assist in the annotation and functional characterization of genes. Functional annotation represents the primary phase for elucidating the function of acquired sequences through BLAST analysis. Conduct a BLAST search within a sequence database to locate similar sequence facilitating the discovery of homologous genes in different species. The subsequent phase involves annotating these sequences process accomplished by merging the gene ontology term. A Phylogenetic tree to create to elucidate the ancestral relationship between heat shock protein (hsp70KDa 1A) and other heat shock protein that are closely related. The construction of phylogenetic tree employ a character based method known as the neighbor joining method, utilizing the Mega11 tool [22], which probability based approach and for construction phylogenetic tree and evolutionary model.

### 2.7 Molecular dynamic simulation (MD)

Molecular dynamics simulations (MD) were operated employing Desmond software from Schrödinger LLC [23] for a duration of 100 ns (ns). During these simulations, receptor-ligand docking was executed to assess the rigid binding interactions of selected compounds with the target protein [24]. The molecular dynamic (MD) analysis was based on Newton's classical equations of motion to evaluate the binding status of the ligands within a physiological environment [25]. The proteins and ligands underwent optimization and minimization using Maestro's Protein Preparation Wizard, which addressed steric clashes, unfavorable contacts, and distorted geometries. The System Builder tool facilitated the construction of the simulation systems, utilizing the TIP3P solvent model—an orthorhombic box—with the OPLS_2005 force field [26]. To neutralize the system, counter ions were introduced and a sodium chloride concentration of 0.15 M was added to replicate physiological conditions at a temperature of 300 K and a pressure of 1 atm throughout the simulation.

## 3 Results

### 3.1 ADMET profiling and toxicity assessment of drug candidates

The web server utilizes canonical simplified molecular input line entry system (SMILEs) is the input data format for molecular prediction with ChemDraw integrated as a molecular editor for canonical simplified molecular input line entry system (SMILEs) generation. The two drug compounds including as (Edelfosine, Ilmofosine) were capitulated from PubChem (https://pubchem.ncbi.nlm.nih.gov/) and the outcomes can be retrieved in the form of CSV file. Each drug molecules, including Edelfosine (16 SMILEs) and Ilmofosine (14 SMILEs) underwent fluorination after being generated from ChemDraw. In the context of ADMET properties, total 30 SMILEs were derived from ChemDraw. An ideal drug candidate exhibits timely absorption and efficient distribution within the system, enabling effective metabolism and action. Toxicity stand as another pivotal factor, frequently taking precedence over ADME characteristics. Furthermore, to assessed the impact of drug fluorination on both normal and tumor cell line by CLC-Pred. To find out the toxicity of all these drug molecules is presented in supplementary (Table 1S). Various transporter has been demonstrated to influence the activities of certain drugs consequently affecting their ADMET properties. The resulting toxicity is summarized as gastric carcinoma, lung carcinoma, non-small cell lung carcinoma, breast adenocarcinoma, colon adenocarcinoma, uterine corpus sarcoma and prostate carcinoma.

**Table 1:** Visualization of best docked heat shock protein (HSP70KDa1A) with fluorinated Edelfosine.

Edelfosine SMILEs	Interaction Residues	Score
O=P([O-])(OCC[N+](C)(C)C)OCC(OC)COCCCCCCCCCCCCCCCCCC(F)(F)F	Asp8, Thr12, Tyr13, Arg34, Thr35, Glu173, Asp197, Gly199, Asp204, Lys269, Arg270, Gly337, Arg340, Asp364	−5.8 kcal/mol
O=P([O-])(OCC[N+](C)(C)C)OCC(OC)COCCCCCCCCCCCCCCCCC(F)(F)C(F)(F)F	Tyr11, Gly10, Tyr13, Asn33, Asp51, Lys69, Asp197, Gly199, Gly200, Thr202, Arg270, Val335, Arg340, Asp364, Val367	−6.6 kcal/mol
O=P([O-])(OCC[N+](C)(C)C)OCC(OC)COCCCCCCCCCCCCCCCC(F)(F)C(F)(F)C(F)(F)F	Asp8, Gly10, Thr11, Thr12, Tyr13, Arg34, Thr35, Lys69, Glu173, Asp197, Gly200, Thr202, Asp204, Arg270, Arg340, Pro363, Asp364, Glu365	−6.5 kcal/mol
O=P([O-])(OCC[N+](C)(C)C)OCC(OC)COCCCCCCCCCCCCCCC(F)(F)C(F)(F)C(F)(F)C(F)(F)F	Asp8, Gly10, Thr11, Thr12, Tyr13, Asn33, Lys69, Asp197, Gly199, Gly200, Thr202, Arg270, Val335, Gly337, Arg340, Asp364, Val367	−7.0 kcal/mol
O=P([O-])(OCC[N+](C)(C)C)OCC(OC)COCCCCCCCCCCCCCC(F)(F)C(F)(F)C(F)(F)C(F)(F)C(F)(F)F	Asp8, Thr12, Tyr13, Asn33, Arg34, Thr35, Glu173, Asp197, Gly200, Thr202, Asp204, Arg270, Arg340, Asp364	−7.5 kcal/mol
O=P([O-])(OCC[N+](C)(C)C)OCC(OC)COCCCCCCCCCCCCC(F)(F)C(F)(F)C(F)(F)C(F)(F)C(F)(F)C(F)(F)F	Asp8, Gly10, Thr11, Thr12, Tyr13, Thr35, Glu173, Gly199, Gly200, Thr202, Asp204, Arg270, Gly336, Gly337, Arg340, Asp364, Glu365	−5.4 kcal/mol
O=P([O-])(OCC[N+](C)(C)C)OCC(OC)COCCCCCCCCCCCC(F)(F)C(F)(F)C(F)(F)C(F)(F)C(F)(F)C(F)(F)C(F)(F)F	Asp8, Thr12, Tyr13, Asn33, Asp51, Lys54, Asn55, Glu173, Asp197, Gly199, Glu266, Arg267, Arg270	−7.1 kcal/mol
O=P([O-])(OCC[N+](C)(C)C)OCC(OC)COCCCCCCCCCCC(F)(F)C(F)(F)C(F)(F)C(F)(F)C(F)(F)C(F)(F)C(F)(F)C(F)(F)F	Asp8, Gly10, Thr11, Thr12, Tyr13, Asn33, Arg34, Lys69, Glu173, Asp197, Gly199, Gly200, Thr202, Asp204, Glu266, Arg270, Gly336, Gly337	−7.6 kcal/mol
O=P([O-])(OCC[N+](C)(C)C)OCC(OC)COCCCCCCCCCC(F)(F)C(F)(F)C(F)(F)C(F)(F)C(F)(F)C(F)(F)C(F)(F)C(F)(F)C(F)(F)F	Tyr13, Asp67, Glu229, Asp232, Arg259, Arg262, Glu266, Arg270, Gly337, Arg340	−6.4 kcal/mol
O=P([O-])(OCC[N+](C)(C)C)OCC(OC)COCCCCCCCCC(F)(F)C(F)(F)C(F)(F)C(F)(F)C(F)(F)C(F)(F)C(F)(F)C(F)(F)C(F)(F)C(F)(F)F	Tyr13, Asn33, Asp51, Lys54, Asn55, Gly200, Glu266, Arg267, Lys269, Arg270, Gly337, Ser338, Arg340, Asp364	−8.0 kcal/mol
O=P([O-])(OCC[N+](C)(C)C)OCC(OC)COCCCCCCCC(F)(F)C(F)(F)C(F)(F)C(F)(F)C(F)(F)C(F)(F)C(F)(F)C(F)(F)C(F)(F)C(F)(F)C(F)(F)F	Asp8, Gly10, Thr12, Tyr13, Asp51,Glu173, Asp197, Gly199, Gly200, Thr202, Glu266, Lys269, Arg270, Gly336, Gly337, Arg340, Asp364	−7.2 kcal/mol
O=P([O-])(OCC[N+](C)(C)C)OCC(OC)COCCCCCCC(F)(F)C(F)(F)C(F)(F)C(F)(F)C(F)(F)C(F)(F)C(F)(F)C(F)(F)C(F)(F)C(F)(F)C(F)(F)C(F)(F)F	Asp8, Gly10, Thr11, Thr12, Tyr33, Asn33, Asp51, Glu173, Asp197, Gly199, Gly200, Asp204, Glu266, Lys269, Arg270, Gly336, Gly337, Ser338, Arg340, Asp364	−8.4 kcal/mol
O=P([O-])(OCC[N+](C)(C)C)OCC(OC)COCCCCCC(F)(F)C(F)(F)C(F)(F)C(F)(F)C(F)(F)C(F)(F)C(F)(F)C(F)(F)C(F)(F)C(F)(F)C(F)(F)C(F)(F)C(F)(F)F	Asp8, Thr12, Thr35, Glu173, Asp197, Gly199, Gly200, Thr202, Arg270, Val335, Asp364, Glu365,	−8.3 kcal/mol
O=P([O-])(OCC[N+](C)(C)C)OCC(OC)COCCCCC(F)(F)C(F)(F)C(F)(F)C(F)(F)C(F)(F)C(F)(F)C(F)(F)C(F)(F)C(F)(F)C(F)(F)C(F)(F)C(F)(F)C(F)(F)C(F)(F)F	Gly10, Tyr13, Asn33, Thr35, Glu173, Gly199, Glu266,Arg267, Lys269, Arg270, Gly337, Ser338, Arg340, Asp364, Glu365	−6.1 kcal/mol
O=P([O-])(OCC[N+](C)(C)C)OCC(OC)COCCCC(F)(F)C(F)(F)C(F)(F)C(F)(F)C(F)(F)C(F)(F)C(F)(F)C(F)(F)C(F)(F)C(F)(F)C(F)(F)C(F)(F)C(F)(F)C(F)(F)C(F)(F)F	Asp8, Gly10, Thr11, Thr12, Thr35, Glu173, Asp197, Gly199, Gly200, Glu266, Arg267, Arg270, Gly337, Arg340, Asp364,	−7.3 kcal/mol
O=P([O-])(OCC[N+](C)(C)C)OCC(OC)COCCC(F)(F)C(F)(F)C(F)(F)C(F)(F)C(F)(F)C(F)(F)C(F)(F)C(F)(F)C(F)(F)C(F)(F)C(F)(F)C(F)(F)C(F)(F)C(F)(F)C(F)(F)C(F)(F)F	Asp8, Gly10, Tyr13, Asn33, Asp51, Gly200, Asp204, Glu266, Arg267, Lys269, Arg270, Val335, Gly336, Gly337, Asp364	−8.2 kcal/mol

### 3.2 Protein receptor selection

The 3D model of the heat shock protein (HSP70KDa1A) was generated through the utilization from 1-click docking server and further obtained from Protein Data Bank (PDB). These structures were assessment via Ramachandran Plot, ERRAT, verify3D and molprobity. The ERRAT score of 95.40 % demonstrate a high level of overall structural quality, while the Verify3D score of 75 % confirms the compatibility of the protein structure with its 3D environment. Additionally, the Ramachandran plot demonstrated that 93 % of the residues fall within the favored regions, further conformational the reliability and accuracy of the protein model for subsequent evaluation as illustrated in (Fig. 1). Conducted energy minimization to refine the geometry and resolve steric clashes with in initial model. The heat shock protein (HSP70KDa1A) was designed through Biovia Discovery Studio.

**Fig. 1:** Validation of the HSP70KDa1A protein structure using (A) ERRAT, (B) Verify3D, and (C) Ramachandran plot confirms its high quality and reliability.

### 3.3 Identification and design of drug ligand

Analog of two-drug ligand select for the ADMET properties, identifying both similarities and differences between Edelfosine and Ilmofosine. Edelfosine is an alkylphosphocholine with exhibit in vitro and in vivo anticancer properties. Ilmofosine is the extensively studies alkylphophocholine recognized for its effectiveness in treating cutaneous metastasis in breast cancer. Both of these drugs possess potent response modulating properties as inhibitors of cancer cell growth. To evaluate the anticancer properties of these drug molecules in both normal and cancerous cells. These drug molecules were chosen on the basis of lower molecular weight. The molecular weight and molecular formula of Edelfosine (523.7, C_27_H_58_NO_6_P) respectively, while Ilmofosine is (525.8, C_26_H_56_NO_5_PS).

### 3.4 Molecular docking

Molecular docking serves as a predictive tool for protein-ligand complex formation, comprising two essential components, a search algorithm responsible for generating potential protein drug complex geometries process known as pose generation and scoring function that evaluate the binding affinity of drug and protein based on the complex geometry. Molecular docking was perform for the assessment of binding interactions of 30 fluorinated drug molecules with the heat shock protein (HSP70KDa1A). The docking finding, highlighted in Table 1, Table 2 that all compounds exhibited strong binding, with the lowest docking scores suggested high binding affinities. The fluorinated Edelfosine and Ilmofosine drugs demonstrated the best possible scores up to −8.4 kcal/mol. The important residues that play a role in binding such as Asp8, Gly10, Thr12, and Arg270. A re-docking was confirmed the consistency of the docking scores and poses. These investigations indicated the significance of these fluorinated drugs as effective inhibitors of heat shock protein (HSP70KDa1A). The figures despite a clear ligand-protein networking from molecular docking simulations. Fig. 2 elaborated the active site of ligand, forming important hydrogen bonds and hydrophobic interactions with potential residues, including Glu and Asn, highlighting a strong binding affinity. Fig. 3 shown an alternative protein conformation with ligand, particularly highlighting unique patterns interaction, such as significant hydrophobic connection. These visualizations collectively underscore the adaptability of the target ligands to different binding sites, supporting our predicted conclusion about the targets potent ligands for enhanced biological activity. The new molecule showed equal or higher binding affinities than known drugs, forming stronger hydrogen bonds and hydrophobic interactions with target proteins. These findings highlighting the new compounds as promising candidates for drug development. The docking scores reflect binding affinities, with lower scores indicating stronger interactions. Notably, the new drugs exhibited significantly lower docking scores than the known drugs, indicating effective and enhanced binding potential and inhibition. Furthermore, specific interactions, such as hydrogen bonds and hydrophobic contacts, support these findings. These results highlights the new compounds as promising drug candidates for further therapeutic evaluation. To establish the accuracy of our inventions a re-docking assessment, which authenticated consistent docking scores and binding poses through various investigation. The 1-Click docking server was exploited for docking and the resulting docking protein structure were visualized using Biovia Discovery Studio (https://discover.3ds.com) and Pymol (https://pymol.org/2/).

**Table 2:** Visualization of best docked heat shock protein (HSP70KDa1A) with fluorinated Ilmofosine.

Ilmofosine SMILEs	Interaction Residues	Score
COCC(COP([O-])(OCC[N+](C)(C)C)=O)CSCCCCCCCCCCCCCCCC(F)(F)F	Asp8, Thr12, Tyr13, Arg34, Thr35, Glu173, Asp197, Gly199, Asp204, Lys269, Arg270, Gly337, Arg340, Asp364	−6.0 kcal/mol
COCC(COP([O-])(OCC[N+](C)(C)C)=O)CSCCCCCCCCCCCCCCC(F)(F)C(F)(F)F	Asp8, Thr12, Tyr13, Arg34, Glu173, Asp197, Gly199, Gly200, Thr202, Asp204, Arg270, Ser338, Arg340, Asp364	−4.9 kcal/mol
COCC(COP([O-])(OCC[N+](C)(C)C)=O)CSCCCCCCCCCCCCCC(F)(F)C(F)(F)C(F)(F)F	Gly10, Thr11, Thr12, Tyr13, Lys69, Glu173, Asp197, Gly199, Gly200, Gly201, Thr202, Arg270, Val335, Gly337, Arg340, Asp364, Val367	−6.5 kcal/mol
COCC(COP([O-])(OCC[N+](C)(C)C)=O)CSCCCCCCCCCCCCC(F)(F)C(F)(F)C(F)(F)C(F)(F)F	Asp8, Gly10, Thr11, Thr12, Tyr13, Lys69, Glu173, Asp197, Gly199, Gly200, Gly201, Thr202, Arg270, Val335, Gly337, Arg340, Val367	−5.5 kcal/mol
COCC(COP([O-])(OCC[N+](C)(C)C)=O)CSCCCCCCCCCCCC(F)(F)C(F)(F)C(F)(F)C(F)(F)C(F)(F)F	Asp8, Gly10, Thr11, Thr12, Tyr13, Asn33, Arg34, Thr35, Asp51, Lys69, Glu173, Asp197, Gly199, Gly200, Thr202, Arg270, Arg340	−7.4 kcal/mol
COCC(COP([O-])(OCC[N+](C)(C)C)=O)CSCCCCCCCCCCC(F)(F)C(F)(F)C(F)(F)C(F)(F)C(F)(F)C(F)(F)F	Asp8, Gly10, Tyr13, Glu173, Asp197, Gly199, Gly200, Arg270, Gly336, Gly337, Arg340, Asp364	−7.7 kcal/mol
COCC(COP([O-])(OCC[N+](C)(C)C)=O)CSCCCCCCCCCC(F)(F)C(F)(F)C(F)(F)C(F)(F)C(F)(F)C(F)(F)C(F)(F)F	Asn33, Arg34, Asp51, Lys54, Asn55, Thr263, Glu266, Arg267, Arg270, Arg340	−5.4 kcal/mol
COCC(COP([O-])(OCC[N+](C)(C)C)=O)CSCCCCCCCCC(F)(F)C(F)(F)C(F)(F)C(F)(F)C(F)(F)C(F)(F)C(F)(F)C(F)(F)F	Asp8, Thr12, Tyr13, Asn33, Arg34, Glu173, Asp197, Gly199, Gly200, Asp204, Arg270, Gly336, Gly337, Arg340, Asp364	−7.1 kcal/mol
COCC(COP([O-])(OCC[N+](C)(C)C)=O)CSCCCCCCCC(F)(F)C(F)(F)C(F)(F)C(F)(F)C(F)(F)C(F)(F)C(F)(F)C(F)(F)C(F)(F)F	Asn33, Asp51, Lys54, Asn55, Glu266, Arg267, Arg270, Arg340, Asp364, Gly365	−6.4 kcal/mol
COCC(COP([O-])(OCC[N+](C)(C)C)=O)CSCCCCCCC(F)(F)C(F)(F)C(F)(F)C(F)(F)C(F)(F)C(F)(F)C(F)(F)C(F)(F)C(F)(F)C(F)(F)F	Asp8, Tyr13, Asn33, Asp51, Lys54, Asn55, Glu173, Asp197, Glu266, Arg267, Arg270, Gly336, Gly337, Arg340	−8.2 kcal/mol
COCC(COP([O-])(OCC[N+](C)(C)C)=O)CSCCCCCC(F)(F)C(F)(F)C(F)(F)C(F)(F)C(F)(F)C(F)(F)C(F)(F)C(F)(F)C(F)(F)C(F)(F)C(F)(F)F	Asp8, Gly10, Thr11, Thr12, Tyr13, Asn33, Asp51, Lys69, Glu173, Asp197, Gly199, Gly200, Thr202, Glu266, Lys269, Arg270, Gly336, Gly337, Arg340, Asp364	−8.4 kcal/mol
COCC(COP([O-])(OCC[N+](C)(C)C)=O)CSCCCCC(F)(F)C(F)(F)C(F)(F)C(F)(F)C(F)(F)C(F)(F)C(F)(F)C(F)(F)C(F)(F)C(F)(F)C(F)(F)C(F)(F)F	Asp8, Gly10, Thr11, Tyr13, Asn33, Arg34, Lys69, Glu173, Asp197, Gly199, Gly200, Thr202, Glu266, Lys269, Arg270, Gly336, Gly337, Ser338, Arg340,	−7.6 kcal/mol
COCC(COP([O-])(OCC[N+](C)(C)C)=O)CSCCCC(F)(F)C(F)(F)C(F)(F)C(F)(F)C(F)(F)C(F)(F)C(F)(F)C(F)(F)C(F)(F)C(F)(F)C(F)(F)C(F)(F)C(F)(F)F	Asp8, Tyr13, Asn33, Pro37, Asp51, Lys54, Asn55, Glu173, Asp197, Gly199, Gly200, Asp232, Glu266, Arg267, Arg270, Gly337, Arg340, Asp364	−8.4 kcal/mol
COCC(COP([O-])(OCC[N+](C)(C)C)=O)CSCCC(F)(F)C(F)(F)C(F)(F)C(F)(F)C(F)(F)C(F)(F)C(F)(F)C(F)(F)C(F)(F)C(F)(F)C(F)(F)C(F)(F)C(F)(F)C(F)(F)F	Asp8, Thr12, Tyr13, Ser14, Arg34, Thr35, Gly199, Gly200, Gly228, Glu266, Lys269, Arg270, Ser273, Gly336, Gly337, Ser338, Arg340, Asp364	−7.2 kcal/mol

**Fig. 2:** Visualization of docked heat shock protein (HSP70KDa1A) binding interaction with fluorinated Edelfosine.

**Fig. 3:** Visualization of docked heat shock protein (HSP70KDa1A) binding interaction with fluorinated Ilmofosine.

### 3.5 Integrated functional annotation and phylogenetic analysis

The structural and functional annotation of heat shock protein (HSP70KDa1A) at both biological and molecular level was executed using Blast2Go. After conducting, a blast search against the total nucleotide sequences of heat shock protein (HSP70KDa1A) to identified and annotated the outcomes that play crucial role in both biological processes and molecular function. Each of these sequences is notable for its significant role at both biological and molecular level, as illustrated in Fig. 4. Blast2Go play a vital role in elucidating the distribution of annotated sequences by incorporation gene ontology (GO) term. Conducted a phylogenetic analysis of heat shock protein (HSP70KDa1A) gene with the objective of validating the conservation of essential domains. The analysis entailed subjecting the nucleotide sequences of heat shock protein (HSP70KDa1A) to blast search against related sequences using the Mega11 tool accessible in the NCBI database. Phylogenetic tree was constructed using various clustering methods to illustrate the significant degree of similarity among species. These trees reveal the evolutionary relationship between species, forming distinct clusters as depicted in Fig. 5.

**Fig. 4:** Functional annotation of heat shock protein (HSP70KDa1A) with GO term distribution.

**Fig. 5:** Phylogenetic tree of heat shock protein (HSP70KDa1A) sequences illustrating evolutionary relationship among species.

### 3.6 Molecular dynamic simulation (MD)

The molecular dynamics simulations of Edelfosine and Ilmofosine determine to heat shock protein (HSP70KDa1A), both run for 100 ns, offered discrimination into their interactions and binding stability. The RMSD evaluation displayed that both complexes concluded equilibrium with the Edelfosine drug complex illustrating higher stability. The protein RMSD in the Edelfosine substantial around 2.0–2.5 Å, while the drug ligand maintained a lower RMSD of 1.0–1.5 Å, denoting strong binding. In comparison, the Ilmofosine drug complex unveiled partially higher RMSD values with the protein stabilizing around 2.5–3.0 Å and the ligand unpredictable between 1.5 and 2.0 Å, indicating a less stable interaction as shown in (Fig. 6, Fig. 7A). The RMSF analysis for both complex identify lowest flexibility in the binding pocket with Edelfosine stabilizing the protein more effectively than Ilmofosine. Moreover, the Ilmofosine complex exhibited enhance flexibility in loop regions, specifically around residues (150–180 and 240–270), denoting localized structural variations as illustrated in (Fig. 6, Fig. 7B). Despite these fluctuations, both drugs maintained the overall secondary structure (SSE) of the heat shock protein (HSP70KDa1A), as sustained by persistent secondary structure elements throughout the simulation as illustrated in (Fig. 6, Fig. 7C). The interaction fraction analysis exposed that both drugs combine with key residues including *TYR 5, ILE 88*, and *ASP 251* though Edelfosine elaborated stronger and more consistent interactions. Hydrophobic interactions dominated the binding for both drug ligands, but Edelfosine exhibit more stable contact with key residues, indicating a stronger affinity for the heat shock protein. In identification, Ilmofosine showed slightly exhausted interactions with fewer hydrogen bonds and lower interaction fractions overall as shown in (Fig. 6, Fig. 7D).

**Fig. 6:** Edelfosine Interaction with heat shock protein (HSP70KDa1A): (A) Shows the root mean square deviation (RMSD) over 100 ns, reflecting protein stability (blue) and ligand fluctuations (red). (B) Depicts the root mean square fluctuation (RMSF) of C-alpha atoms, indicating residue flexibility. (C) Presents the percentage of secondary structure elements (SSE) included, confirming that Edelfosine maintains protein integrity. (D) Highlights the interaction fraction with key residues, emphasizing significant binding interactions.

**Fig. 7:** Ilmofosine Interaction with heat shock protein (HSP70KDa1A): (A) Shows the root mean square deviation (RMSD) over 100 ns, reflecting protein stability (blue) and ligand fluctuations (red). (B) Depicts the root mean square fluctuation (RMSF) of C-alpha atoms, indicating residue flexibility. (C) Presents the percentage of secondary structure elements (SSE) included, confirming that Edelfosine maintains protein integrity. (D) Highlights the interaction fraction with key residues, emphasizing significant binding interactions.

#### 3.6.1 Hydrogen bond analysis

The Edelfosine heat shock protein (HSP70KDa1A) complex determined potent and stable hydrogen bond interaction frequently conserving approximate (320–350) hydrogen bonds throughout the simulation duration. This stability illustrate a strong compatibility and extended engagement between Edelfosine and protein, offering that Edelfosine capably stabilizes the protein configuration through enduring interactions as shown in (Fig. 8A). In distinction, the Ilmofosine complex exhibit a more dynamic hydrogen-bonding pattern, with fluctuating bond computation that reached a maximum of 340 bonds but frequently dropped below 300. This flexibility manifest that Ilmofosine may engage in more transient interactions with the protein, potentially considerate its binding stability and offering a less effective stabilization of the protein structural integrity as illustrated in (Fig. 8D).

**Fig. 8:** (A,D) illustrate hydrogen bond interactions over 100 ns, showing Edelfosine more stable binding compared to Ilmofosine. (B,E) represent the radius of gyration, indicating that Edelfosine induces less structural fluctuation in heat shock protein (HSP). (C,F) show the solvent-accessible surface area (SASA), with Edelfosine maintaining more consistent protein conformation than Ilmofosine.

#### 3.6.2 Radius of gyration (Rg)

The radius of gyration for the Edelfosine determine protein revealed a continuous enhance stabilizing between (21.6–22.0 Å). This trend signify a moderate structural amplification upon ligand binding, which may reflect the drug ligands effective combination into the protein active site. In comparison, the Rg for the Ilmofosine complex showed higher fluctuations ranging between (21.2–21.8 Å), denotive of enhanced configurational flexibility and potential modification compared to Edelfosine as illustrated in (Fig. 8B,E).

#### 3.6.3 Solvent accessible surface area (SASA)

The SASA for Edelfosine remained approximately stable around (17500–18000 Å^2^), displaying a compatible protein conformation and reliable solvent exposure throughout the simulation. In contrast, the SASA for Ilmofosine exhibit more distinct fluctuations alternating between (17000–18000 Å^2^), suggesting greater dynamic variations in the protein structure and emphasizing the potential for less stable binding interactions as shown in (Fig. 8C,F).

## 4 Discussion

Recent studies have focused a lot of emphasis on the ADMET and anti-neoplastic properties of fluorinated phospholipid analogs, particularly Miltefosine, Edelfosine and Ilmofosine. Notably, Edelfosine manufactured alkyl-lysophospholipid has shown that it can cause apoptosis in a variety of cancer cell lines. Ilmofosine another synthetic alkylphosphocholine has also shown promise in preclinical research as an antineoplastic drug. In order to determine these compounds' potential as anti-cancer drugs, it is critical to examine their ADMET profiles. Absorption, distribution, metabolism, excretion and toxicity or ADMET as it known are important factors to take into account while developing new medications. These analyses allow researchers to evaluate a compound's safety and efficacy in vivo as well as its pharmacokinetic and pharmacodynamics properties.

Many studies have carefully examined the ADMET profiles of these fluorinated phospholipid analogs, providing insightful information on their potential as anti-cancer drugs. For example, a study by Refs. [27,28] examining Miltefosine pharmacokinetics in several animal models found that it has beneficial properties, such as substantial oral bioavailability and extensive tissue distribution. These results make it a good option for additional study in clinical trials. Similarly, a study by Ref. [29] Edelfosine had a positive pharmacokinetic profile and indicated good tolerance in mice. Research studies have examined these substances antineoplastic potential in addition to evaluating their ADMET profiles [30]. For instance, a study by Ref. [31] Ilmofosine was discovered to have potent anticancer effect against the particularly aggressive form of brain cancer known as glioblastoma multiform. Another study by Ref. [32] Miltefosine promoted apoptosis and inhibited autophagy, which prevented human pancreatic cancer cells from proliferating. An essential phase in the discovery of new antineoplastic drugs is evaluating the ADMET and antineoplastic profiles of fluorinated phospholipid analogs like Edelfosine and Ilmofosine. Our exploration intimate that fluorinated ALPs hold considerable capability for improving current medications by increasing the stability of compounds and biological activity. Fluorine substitution may enhance membrane absorbent reduce biodegradation and increase binding interactions with beneficial targets. Consequently, fluorinated ALPs could extend emphasized efficiency compared to non-fluorinated portraits potentially manipulating the limitations of current medication strategies and extend a narrative approach for drug improvement. Although there remains much to learn about the pharmacokinetic and pharmacodynamics properties of these substances, the knowledge gained from recent research investigations suggests they have a significant potential as anti-cancer medicines, suggesting more investigation [33].

The primary objective of this study was to find drugs with ADMET profiles that were both similar to and distinct from those of the original medications Edelfosine and Ilmofosine. Additionally, we aimed to evaluate the interactions of selected drug analogs using molecular docking with heat shock protein (HSP70KDa 1A/1B) as well as the activity of each drug derivative against both normal and malignant cell lines. In the field of drug research and development, analyzing the ADMET profiles of these medications is crucial because it includes important elements including absorption, distribution, metabolism, excretion and toxicity. PubChem provided the two drug compounds Edelfosine and Ilmofosine. ChemDraw was used to extract 30 SMILEs notations for the evaluation of the ADMET characteristics. An important component toxicity frequently takes precedence over ADMET considerations. Additionally, the toxicity of these medications was estimated using CLC-Pred to identify the effect of fluorination on normal and malignant cell lines. All pharmacological compounds hazardous effects were examined in light of the possibility that specific transporters could affect drug actions and in turn have an impact on ADMET characteristics [34]. Uterine corpus sarcoma, colon adenocarcinoma, non-small cell lung carcinoma, papillary renal carcinoma, lung carcinoma, breast adenocarcinoma, prostate carcinoma and stomach carcinoma are among the toxicity that have been condensed. The effectiveness of each drug derivative against both normal and tumor cell lines was examined and used molecular docking to look at how particular drug analogs interacted with a heat shock protein. The proliferation of cancer cells is inhibited by the powerful biological responses that Edelfosine and Ilmofosine modulate. These pharmacological compounds were chosen based on molecular weight criteria after their anticancer effects were evaluated in both cancer and normal cells. The molecular weight and molecular formula of Edelfosine (523.7, C_27_H_58_NO_6_P) and Ilmofosine (525.8, C_26_H_56_NO_5_PS). Additionally, we used molecular docking to investigate how particular drug analogs interacted with heat shock protein (HSP70KDa 1A).

The molecular dynamics simulations (MD) distribute defining insight into the confining dynamics of Edelfosine and Ilmofosine drugs with heat shock protein (HSP70KDa1A) identify consequential alteration in their interaction profile. Edelfosine indicate enhanced binding stability interpreted by lower root mean square deviation (RMSD) scores, which ranged from (2.0–2.5 Å) for the protein and (1.0–1.5 Å) for the drug ligand associated a strong and reliable complex configuration. This stability is additional supported by enduring hydrogen bond complex preserving approximately (320–350) hydrogen bonds throughout simulation, which confirm the notion that Edelfosine drug adequately stabilizes the protein configuration. In distinction, Ilmofosine drug unveiled higher RMSD values (2.5–3.0 Å for the protein and 1.5–2.0 Å for the drug ligand) and greater fluctuations in both radius of gyration and solvent-accessible surface area, implying less stable interactions and higher compositional flexibility [34]. In this study, conducted a 100 ns molecular dynamics (MD) simulation of the 3LQ8 protein with ligands H06, H12, H30, H36, and Foretinib. The investigation describe that all complexes performed stability after approximately 20 ns with average RMSD values ranging from (1.790–2.420 Å), suggesting stable configuration. These findings are consistent, who reported similar RMSD values for cyclohexane-1,3-dione derivatives, highlighting stable ligand-protein interactions. RMSF analysis revealed average values between (0.879–1.112 Å), indicating less fluctuations and greater stability aligning with the results. Minimum fluctuations were showed in residues outside the active sites, likely due to their flexible nature [[35], [36], [37]]. Protein and drug ligand contact dynamics demonstrate key interactions, such as hydrogen bonds and hydrophobic interactions, essential for maintaining stability throughout the simulation. The results corroborate those, who observed similar interaction profiles, emphasizing the significance of specific amino acid residues in ligand binding. We also analyzed ligand properties, such as radius of gyration and solvent-accessible surface area indicating high stability within the protein pocket. Overall, MD simulation findings align with existing literature reinforcing their relevance in drug design and the development of therapeutic agents. These detections involve that Edelfosine drug binding affinity may contribute to its therapeutic capability, probably increasing its function in regulation stress response pathways indication in cancer progression, considering that the less stable binding of Ilmofosine could limit its effectiveness as a therapeutic agent. Through stabilizing carcinogenic substrate proteins, the molecular chaperone 70KDa1A aids in the survival and proliferation of cancer cells. For cancer therapy, targeting and inhibiting 70KDa1A have shown promise. These results are consistent with other studies that showed the anticancer efficacy of HSP90 inhibitors, such as Miltefosine and its analogs [[38], [39], [40]].

## 5 Conclusions

This study identified two drug analogs exhibiting ADMET profile to those of the original drugs and assessed their activity on both normal and cancerous cell line. Additionally, we explored their potential as inhibitor of heat shock protein (HSP70KDa1A) through molecular docking analysis. These findings provide a basis for subsequent experimental validation and refinement of these drugs analogs as prospective anticancer agents. This study includes further experimental validation of the identified analogs, exploration of their efficacy in animal models and investigation of potential drug-drug interactions with commonly prescribed medications. Novel compounds with superior binding affinities compared to known drugs, suggesting their potential as effective therapeutic candidates. The molecular dynamics simulations unveil that Edelfosine drug display dominating binding stability to heat shock protein analyze to Ilmofosine, identified by lower RMSD values and reliable hydrogen bond complex. These finding indicates that Edelfosine drug may be a highly effective therapeutic retardation, while Ilmofosine drug less stable interaction demonstrate diminished capability for maximum therapeutic Consequence. This study highlight the characteristics of consideration drug binding features to inform the evolution of effective therapies targeting heat shock protein dysregulation in cancer and related diseases. Additionally, future studies could focus on the development of new drug derivatives based on the identified compounds and their further optimization for improved ADMET properties and activity against tumor cell lines. Finally, it would be beneficial to explore the potential of these compounds for use in combination therapy with other anticancer agents to enhance their therapeutic efficacy.

## CRediT authorship contribution statement

**Saqib Ishaq:** Writing – original draft, Software, Data curation, Conceptualization. **Obaid Habib:** Writing – original draft, Software, Formal analysis, Data curation, Conceptualization. **Abdul Aziz:** Validation, Supervision, Methodology, Investigation, Formal analysis. **Raheel Tahir:** Visualization, Validation, Resources, Investigation, Formal analysis. **Hira Mushtaq:** Visualization, Validation, Investigation, Data curation. **Said Hassan:** Software, Resources, Investigation, Formal analysis. **Sarah Sarwar:** Software, Resources, Investigation, Data curation. **Mohammad S. Mubarak:** Writing – review & editing, Visualization, Formal analysis. **Ajaz Ahmad:** Writing – review & editing, Resources, Project administration, Funding acquisition. **Amin Ullah:** Writing – review & editing, Validation, Investigation, Funding acquisition, Formal analysis.

## Informed consent statement

No.

## Data availability statement

The datasets used in this study are publicly available in the PubChem database. The drugs Edelfosine (https://pubchem.ncbi.nlm.nih.gov/#query=edelfosine) and Ilmofosine (https://pubchem.ncbi.nlm.nih.gov/#query=ilmofosine) were retrieved from this database.

## Institutional review board statement

Not applicable.

## Funding

The author did not receive any funding.

## Declaration of competing interest

The authors declare the following financial interests/personal relationships which may be considered as potential competing interests:Amin ullah reports financial support was provided by Iqra national university Peshawar. Ajaz Ahmad reports a relationship with 10.13039/501100002383King Saud University that includes: employment and funding grants. Amin Ullah has patent n/a pending to n/a. No potential conflict of interest. If there are other authors, they declare that they have no known competing financial interests or personal relationships that could have appeared to influence the work reported in this paper.
